# Role of microvascular endothelial cells on proliferation, migration and adhesion of hematopoietic stem cells

**DOI:** 10.1042/BSR20192104

**Published:** 2020-03-20

**Authors:** Fanli Lin, Shuyue Wang, Hao Xiong, Yang Liu, Xiaoming Li, Chunlan Huang

**Affiliations:** 1 Department of Hematology, Affiliated Hospital of Southwest Medical University, Luzhou, Sichuan, China; 2 The affiliated hospital of Panzhihua University, Panzhihua, Sichuan, China; 3 Stem Cell Laboratory and Department of Hematology, Affiliated Hospital of Southwest Medical University, Luzhou, Sichuan, China

**Keywords:** Cell adhesion, Cell migration, Cell proliferation, Chemotaxis, Hematopoietic stem cells, Microvascular endothelial cells

## Abstract

**Background:** The present study investigated the effects of microvascular endothelial cells (MECs) on the chemotaxis, adhesion and proliferation of bone marrow hematopoietic stem cells (HSCs) *ex vivo*. **Methods and Results:** MECs were collected from the lung tissue of C57BL/6 mice, and HSCs were isolated with immunomagnetic beads from bone marrow of GFP mice. MECs and HSCs were co-cultured with or without having direct cell–cell contact in Transwell device for the measurement of chemotaxis and adhesion of MECs to HSCs. Experimental results indicate that the penetration rate of HSCs from the Transwell upper chamber to lower chamber in ‘co-culture’ group was significantly higher than that of ‘HSC single culture’ group. Also, the HSCs in co-culture group were all adherent at 24 h, and the co-culture group with direct cell–cell contact had highest proliferation rate. The HSC number was positively correlated with vascular endothelial growth factor (VEGF) and stromal cell-derived factor-1 (SDF-1) levels in supernatants of the culture. **Conclusions:** Our study reports that MECs enhance the chemotaxis, adhesion and proliferation of HSCs, which might be related to cytokines SDF-1 and VEGF secreted by MECs, and thus MECs enhance the HSC proliferation through cell–cell contact. The present study revealed the effect of MECs on HSCs, and provided a basis and direction for effective expansion of HSCs *ex vivo*.

## Introduction

Hematopoietic stem cell (HSC) is a type of adult stem cells, whose self-renewal, maintenance, apoptosis and motional migration are tightly regulated. Most HSCs are in quiescent state under homeostasis, and cycle infrequently for self-renewal or to differentiate into multipotent progenitors (MPPs) and more committed progenitors, with limited self-renewal potential. Hematopoiesis is carefully regulated by both extrinsic and intrinsic mechanism(s), which balance quiescence, self-renewal and differentiation to support normal multi-lineage reconstitution [1–3]. In 1978, Ray Schofield first introduced the important regulatory role of bone marrow niche for HSCs. Since then, the development of experimental techniques and methods have enabled the study of the structural biology of niche, the specific function of different niche components and their roles in the progress of blood diseases. It has been evident that the bone marrow niche can be mainly categorized as the endothelium niche and the perivascular niche. With the continuous improvement of experimental methods and modern equipment, the cellular composition of the bone marrow niche can be clearly identified. Mesenchymal stem cells (MSCs) and endothelial cells (ECs) are the two major types of cells in bone marrow niche. It has been reported that ECs provide a nutrient-rich hematopoietic niche for HSC, which can effectively promote HSC proliferation and differentiation [4–10].

The specific microenvironment for the survival of HSCs is termed as ‘niche’ [11,12]. Scientists have done extensive research on the mechanisms of their maintenance and the complex molecular and cellular composition, but the factors that currently regulate HSCs regulation are still poorly understood. In particular, the role and regulation of perivascular niche in the microenvironment of HSCs is obscure. The present study aims to further examine the effect of ECs on HSCs and explore new approaches to effectively amplify the HSCs *ex vivo*. It has been reported that the lungs also have the function of hematopoietic regulation, and the microvascular endothelial cells (MECs) are the most abundant cells in lung tissue [13]. Therefore, the present study would select mouse lung tissue culture of MECs, and aimed to co-culture with HSCs *ex vivo* to explore the effect of MECs on HSCs, and the mechanisms by which MECs regulate HSCs.

## Materials and methods

### Experimental materials

DMEM-F12, and typsin medium was purchased from Hyclone (U.S.A.). Fetal bovine/calf serum (FBS) and bovine serum albumin (BSA) powder were purchased by Nanjing Sansheng Biological Company (China). The mouse Ficoll lymphocyte separation solution was purchased from Tianjin TBD (China). Mini MACS CD117 cell sorting kit was purchased from Miltenyi Biotec (Germany). Mouse vascular endothelial growth factor (VEGF) was purchased from ACRO Biosystems (China). Type I collagenase and gelatin dry powder were purchased from Sigma (U.S.A.). Mouse IL-3 and mouse stem cell growth factor were purchased from Novus Corporation (U.S.A.). APC rat Anti-Mouse CD117, rat IgG Isotype control APC, PE rat Anti-Mouse CD34 and Rat IgG Isotype control PE were purchased from BD Corporation (U.S.A.).

### Experimental animals

C57BL/6 wild-type mice and green fluorescent protein (GFP) transgenic mice were purchased from the Experimental animals company of Dashuo (Chengdu, China). All mice were bred in-house in a pathogen-free mouse facility room. Mice of 4–6 weeks of age (15–25 g) were anesthetized with 0.3% sodium phenobarbital solution (0.1 ml/10g; i.p.) and killed by cervical dislocation method. In brief, the root of the mouse tail was hold with the right hand and lift it up. It was then placed on the squirrel cage cover or other rough surface. The mouse head and neck were pressed down with left thumb and index finger. The cervical spine was dislocated, and the spinal cord was disconnected from the brain stem, for which the experimental animals died immediately. Animal experiments were performed in accordance with guidelines approved by the Institutional Animal Care and Use Committee (IACUC) at the Southwest Medical University in China.

### Microvascular endothelial cell culture

Four- to six-week-old C57BL/6 wild-type mice were killed and whole-lung tissue was obtained. The cells obtained by digestion process were cultured in DMEM-F12 medium containing 10% FBS, 1% cyan-streptomycin, and 2 ng/ml VEGF. Cells were placed in a six-well plate pre-coated with gelatin and cultured in a 37°C, 5% CO_2_, 95% humidity incubator. After 10–14 days, the cells grew into a “paving stone like” for use.

### Immuno-magnetic bead sorting CD117+ HSCs

Four- to six-week-old GFP mice (C57BL/6 line) were killed, and after cervical spinal cord dissection, the bone marrow cells were washed out from tibia and femur using a mouse Ficoll lymphocyte separation solution to obtain monocytes (MNC) by density gradient centrifugation.

### The chemotaxis of MEC to HSC

Using 5 µm Transwell equipment, HSCs were placed in the Transwell upper chamber at a density of 4 × 10^4^ per well, and MECs in the lower chamber at a density of 2 × 10^4^ per well. The control group was set, and the number of HSCs penetrating from the upper chamber to the lower chamber for 24 h was counted separately.

### The adhesive attraction of MEC to HSC

The MECs were seeded into the 96-well plate at a density of 10^4^ per well, and the HSCs were seeded into the plate at a density of 10^4^ per well after the MECs were attached. The number of suspension cells in each group were counted at 1, 6, 12, 18 and 24 h.

### The effects of MECs on HSCs proliferation under different culture modes

The MECs were seeded in lower chambers of Transwell (0.4 μm) and 24-well plates respectively in at a density of 10^4^/well, meanwhile, HSCs were seeded in upper chamber and on a confluent MECs layer respectively at a density of 10^4^/well at 37°C in 5% CO_2_. Cells were suspended in DMEM-F12 medium containing 10% FBS, 1% cyan-streptomycin, 25 ng/ml mouse stem cell growth factor (SCF) and 25 ng/ml mouse interleukin 3 (IL-3). Then, the cell counting and CCK-8 methods were used to detect the proliferation of HSCs in each group on the day 1, 3, 5 and 7 of cell culture. And flow cytometry was used to detect the change of CD117^+^ CD34^+^ HSC ratio before and after amplification in the co-culture group.

### Detection of SDF-1 and VEGF expressions by ELISA

The MECs were seeded in lower chambers of Transwell (0.4 μm) and 96-well plates respectively at a density of 3 × 10^4^/well, while HSCs were seeded in upper chamber and on a confluent MECs layer respectively at a density of 1.5 × 10^4^/well at 37°C in 5% CO_2_. The expression levels of SDF-1 and VEGF on day 1, 3, 5 and 7 of each group were detected by ELISA.

### Statistical analysis

Data are expressed as the mean ± standard deviation (SD). The one-way analysis of variance (ANOVA) with one-tailed unpaired *t*-tests were used to compare the data between the two groups, by using Graphpad prism 6.0 software. *P* < 0.05 was considered as a statistically significant difference. The correlation between SDF-1 and VEGF in different groups were assessed using Spearman correlation analysis. Correlation analyses were performed using SPSS 19.0 software.

## Results

### The morphology of microvascular endothelial cell

The primary cell of MEC began to be adherent after 6 h of culture and fully attached after 24 h. On day 3, the cells began to aggregate and grow to form a cell cluster with uniformed morphology (Figure 1A). On day 6, the pseudopods of adjacent cells began to fuse (Figure 1B), and day 10–14 cells grew to 80% fuse, showing a “paving stone-like” appearance (Figure 1C,D). We used flow cytometry to examine the purity of MEC. The expression rate of immunophenotype vWF was 81.39%, CD31 expression rate was 45.8%, CD34 expression rate was 57.48% and CD45 expression rate was 0.17% (Figure 1E), which is in line with the phenotypic characteristics of MEC [14–17].

**Figure 1:** The morphology and flow identification of MECs (**A**) MEC forms for 3 days (×100); (**B**) MEC forms for 6 days (×100); (**C**) MEC forms for 10 days (×100); (**D**) MEC forms for 14 days (×100), showing a “paving stone-like” appearance; (**E**) on day 8 of MECs culture, identification of MECs CD34, CD45, CD31 and vWF expression by flow cytometry.

### MEC not affects HSC differentiation

Flow cytometric analysis identified the CD117^+^HSC sorted by flow cytometry with a purity of 99.51%. In this experiment, the co-expression rate of the selected HSCs markers CD117^+^ and CD34^+^ was 75.85%. After co-culture with MEC for 7 days, the co-expression rate of HSC markers CD117^+^ and CD34^+^ was 92.06%, indicating that the suspension cells collected after co-culture with MEC were still HSCs with differentiation potential, and promoted the expression of CD34 during co-culture (Figure 2).

**Figure 2:** Identification of HSC phenotype during cell culture (**A**) Flow cytometric analysis of HSC CD117 and CD34 expression before co-culture with MECs. (**B**) After 7 days co-culture with MECs, HSC CD117 and CD34 expression were analyzed by flow cytometric again.

### MEC facilitates HSC migration

After 24 h of cell culture, the penetration rate of HSCs from the transwell’s upper chamber to the lower chamber in the co-culture group were significantly increased compared with the HSC group (4.870% ± 0.503% vs 1.643% ± 0.134%, *n* = 5, *P* < 0.001), and the lower chamber GFP-labeled cells (i.e., HSCs) were also significantly increased compared with the simple HSC group when observed under fluoroscopy (Figure 3A,B).

**Figure 3:** Chemotaxis and Adhesion of HSC by MEC (**A**) When co-cultured with MECs for 24 h, GFP-labeled cells (i.e. HSCs) in the lower chamber of transwell in fluorescence microscope. (**B**) GFP-labeled cells in fluorescence microscope at 24 h of HSC group. (**C**) Comparison of the adhesive attraction of MEC on HSC. Adhesion rate of HSCs at 1 h in the co-culture group increased significantly compared with the HSC group (*n*=3, *P<0.05).

### MEC facilitates HSC attraction

We found that the Adhesion rate of HSCs in the co-culture group at 1, 6, 12, 18 and 24 h were higher than that in the HSC group. Among them, this difference is most obvious at 1 h (20% ± 5% in the co-culture group vs 5% ± 1.8% in the HSC group, *n* = 3, *P* < 0.05). At 24 h, the adhesion rate of the co-culture group was 90% ± 6%; however, which is 78.3% ± 7.6% in the HSC group due to gravity (Figure 3C).

### There are different effects of MEC on HSC proliferation under different culture modes

The counting of HSCs in three groups were increased during the culture (Figure 4A). In order to compare the number of HSCs in different groups, cell counting and CCK-8 experiments were used. The HSC proliferation in the 2-D group (i.e. contact culture group) was higher than that in the transwell group (i.e. non-contact co-culture group) and the HSC group(i.e., control group), and which was higher in the transwell group than that in the HSC group (Figure 4B–D): for example, on day 5: the count of HSCs 82.7 ± 11.122 in the 2-D group vs 23.97 ± 7.001 in the transwell group vs 6.138 ± 0.485 in the HSC group (*n* = 5, *P* < 0.0001) and on day 7: the count of HSCs 158.4 ± 8.576 in the 2-D group vs 31.9 ± 2.568 in the transwell group vs 8.8 ± 0.447 in the HSC group (*n* = 5, *P* < 0.0001). In addition, on day 3 of 2D group and the transwell group, HSCs entered the logarithmic growth phase, which were earlier than the fifth day of control group (Figure 4C).

**Figure 4:** Cell proliferation status (**A**) Changes of GFP-labeled cells in Fluorescent microscopy of different groups at different times (×100)**.** From 1 to 7 days, the number of GFP-labeled cells in the three groups was gradually increased, and the proliferation of 2-D group was the most obvious. (**B**) Comparison of cell yields of cultivation of three groups at different times (*n*=5, *^a^P*<0.05 vs HSC group; *^b^P*<0.05 vs Transwell group). (**C**) The growth curve of HSCs in three groups (*n*=5, *P<0.05, ^##^*P*<0.001). (**D**) Cell proliferation analysis by CCK-8 (*n*=3, ^##^*P*<0.001).

### MEC secretes SDF-1 and VEGF to promote HSC proliferation

To investigate the effect of cytokines on proliferation of HSCs, SDF-1 and VEGF were determined by ELISA. As shown in Figure 5, SDF-1 was more highly expressed in the 2-D group and Transwell group than HSC group or MEC group (109.529 ± 1.503 in the 2-D group and 91.678 ± 3.190 in the Transwell group vs 32.509 ± 1.487 in the HSC group (*n* = 5, *P* < 0.001) and 55.697 ± 4.146 in the MEC group (*n* = 5, *P* < 0.001). We also found a higher concentration of VEGF in 2-D group and Transwell group than HSC group or MEC group (84.649 ± 3.074 in the 2-D group and 76.061 ± 2.951 vs 25.410 ± 1.417 in the HSC group (*n* = 5, *P* < 0.001) and 41.043 ± 1.907 in the MEC group (*n* = 5, *P* < 0.001). In addition, Correlation analysis between the number of HSCs and SDF-1 and VEGF contents showed that the number of HSCs was highly positively correlated with the levels of SDF-1 and VEGF in the cell culture supernatant (*P* < 0.001).

**Figure 5:** The supernatant of SDF-1 levels (**A**) and VEGF levels (**B**) by ELISA in each group (*n*= 3, *^a^P<*0.05 vs HSC group; *^b^P<* 0.05 vs MEC group)

## Discussion

It is difficult to obtain continuous expansion of pluripotent progenitor cells in liquid suspension culture in studies in vitro. However, when hematopoietic progenitor cells are co-cultured with stromal cells and matrix-derived factors, relatively longer-lasting amplification can be obtained [18]. It was reported that highly purified mouse CD117^+^ HSCs can achieve more efficient proliferation in the presence of microenvironment contain of microvascular endothelial cells. Davis et al. [19] demonstrated the role of endothelial cells in stimulating the proliferation of HSCs. They co-cultured Porcine microvascular endothelial cells (PMVEC) and combined cytokines (GM-CSF, IL-3, SCF, IL-6) with purified human CD34 + bone marrow cells *in vitro*, and observed that in 7 days of culture, the direct contact culture of HSCs with PMVEC monolayers achieved maximum expansion compared to non-contact culture and liquid suspension culture HSCs, and CD34+ hematopoietic stem/progenitor cells were expanded 12.6 times in culture. On the seventh day of cell culture in this experiment, the number of HSCs in the co-culture group (HSCs and microvascular endothelial cells in 2-D) was 41.6 times higher than that in the first day, which was significantly increased compared with Transwell non-contact co-culture group and HSCs culture group. In our study, the expansion of HSCs on the seventh day of the Transwell group was significantly higher than the hematopoietic stem cells alone group, suggesting that cytokines secreted by microvascular endothelial cells might promote the proliferation of HSCs.

In the hematopoietic stem cells microenvironment, HSCs are regulated by a variety of chemokines, cytokines, adhesion molecules and other signals, promoting HSCs colonized in this microenvironment, and in the steady state of self-renewal, proliferation and differentiation [20]. Endothelial cells can promote HSC proliferation and differentiation through a paracrine mechanism, where endothelial cells maintain the survival and self-renewal of HSCs by secreting stromal-derived factor 1 (SDF-1) and binding to the hematopoietic stem cell surface receptor CXCR-4. *In vitro* experiments by Lataillade et al. [21] confirmed that SDF-1 can induce the proliferation of CD34+ stem/progenitor cells, which is consistent with in the present study that the positive correlation between SDF-1 expression and HSCs proliferation (*P* < 0.001). In addition, SDF-1 can promote the secretion of VEGF by endothelial cells, and further promote the proliferation of HSCs. Chi et al. [22] used endothelial cells and HSCs for co-culture *in vitro*, and detected the concentration of VEGF cytokines in the cell culture supernatant by ELISA. The results showed that the expression of VEGF in the co-culture group clearly increased than that in the control group. The 7th day results in our experiment showed that the expression of VEGF was significantly increased in MEC and HSC 2-D contact culture group compared with HSC culture group and Transwell non-contact co-culture group, and the expression of VEGF was positively correlated with the proliferation of HSC, which was consistent with the results of the above mentioned studies. In addition, in this experiment, MECs were directly exposed to HSCs for seven days, HSCs expansion (41.568 times) was significantly increased compared with non-contact co-culture group (11.58 times) and HSC group (4.9 times). It is speculated that in addition to the promotion of HSC proliferation by cytokines secreted by microvascular endothelial cells, cell–cell contact mediated by specific adhesion molecules also plays an important role.

HSC in peripheral blood is regulated by SDF-1, bioactive phosphosphingolipids sphingosine-1-phosphate (S1P) and ceramid-1-phosphate (C1P), and chemokines such as extracellular nucleotides ATP and UTP effectively homing HSC to bone marrow (BM) and adhering through HSC to EC, followed by implantation, and finally repopulation in BM [23]. To promote HSCs proliferation and maintain its regeneration by endothelial cells expressing Notch ligand jagged and transmembrane protein Delta-like [24]. Currently, SDF-1 is the most potent chemotactic agent for HSC, and SDF-1 is a member of the CXC chemokine family and the ligand is CXCR4. SDF-1-induced trans-endothelial behavior is positively correlated with HSC/HPC surface CXCR4 density. SDF-1 also induces the interaction of integrin VLA-4 and LFA-1 with its corresponding endothelial cell ligand vascular cell adhesion molecule 1 (VCAM-1) and intercellular cell adhesion molecule-1 (ICAM-1), promoting the HSCs firmly adheres to the endothelium and eventually through the endothelial cell barrier settles into the “niche” of the bone marrow stroma, rebuilding the host’s hematopoietic function. Greenbaum et al [25]. found that the removal of CXCL12 in Tie-2+ endothelial cells, the number of HSCs in the bone marrow decreased without inducing HSCs mobilization, indicating that endothelial cells play an indispensable role in the survival of HSCs by producing these micro-niche factors.

In conclusion, our study reports that MECs regulate the chemotaxis, adhesion and proliferation of HSCs, which might be related to the role of cytokines such as SDF-1 and VEGF secreted by MEC and the regulation of HSC proliferation through cell–cell contact, which revealed the effect of MECs on HSCs, and provided a basis and direction for effective expansion of HSCs *ex vivo*.

## Abbreviations

EC: endothelial cell
HSC: hematopoietic stem cell
MEC: microvascular endothelial cell
MPP: multipotent progenitor
SDF-1: stromal cell-derived factor-1
VEGF: vascular endothelial growth factor
